The article "Estimation of Response Functions Based on Variational Bayes Algorithm in Dynamic Images Sequences" was retracted in 2017. Reasons: plagiarism; duplicate publication; overlap with other authors' work; overlap with earlier publications.

# Estimation of Response Functions Based on Variational Bayes Algorithm in Dynamic Images Sequences

**DOI:** 10.1155/2016/4851401

**Published:** 2016-08-18

**Authors:** Bowei Shan

**Affiliations:** School of Information Engineering, Chang'an University, Shaanxi 710064, China

## Abstract

We proposed a nonparametric Bayesian model based on variational Bayes algorithm to estimate the response functions in dynamic medical imaging. In dynamic renal scintigraphy, the impulse response or retention functions are rather complicated and finding a suitable parametric form is problematic. In this paper, we estimated the response functions using nonparametric Bayesian priors. These priors were designed to favor desirable properties of the functions, such as sparsity or smoothness. These assumptions were used within hierarchical priors of the variational Bayes algorithm. We performed our algorithm on the real online dataset of dynamic renal scintigraphy. The results demonstrated that this algorithm improved the estimation of response functions with nonparametric priors.

## 1. Introduction

Highly rapid development of machine learning technique offers an opportunity to obtain information about organ function from dynamic medical images, instead of invasive intervention. The unknown input function can be obtained by deconvolution of the organ time-activity curve and organ response function. Typically, both the input function and the response functions are unknown. Moreover, the time-activity curves are also not directly observed since the recorded images are observed as superposition of multiple signals. Analysis of the dynamic image sequences thus require to separate the original sources images and their weights over the time forming the time-activity curves (TACs). The TACs are then decomposed into input function and response functions. Success of the procedure is dependent on the model of the image sequence.

The common model for dynamic image sequences is the factor analysis model [1], which assumes linear combination of the source images and TACs. Another common model is that TAC arises as a convolution of common input function and source-specific kernel [2, 3]. The common input function is typically the original signal from the blood and the role of convolution kernels varies from application area: impulse response or retention function in dynamic renal scintigraphy [4]. In this paper, we will refer to the source kernels as the response functions; however other interpretations are also possible.

Analysis of the dynamic image sequences can be done with supervision of experienced physician or technician, who follows recommended guidelines and uses medical knowledge. However, we aim at fully automated approach where the analysis fully depends on the used model. The most sensitive parameter of the analysis is the model of the response functions (i.e., the convolution kernels). Many parametric models of response functions have been proposed, including the exponential model [5] or piecewise linear model [6, 7]. An obvious disadvantage of the approach is that the real response function may differ from the assumed parametric models. Therefore, more flexible classes of models based on nonparametric ideas were proposed such as averaging over region [8], temporal regularization using finite impulse response filters [9], or free-form response functions using automatic relevance determination principle in [10].

The article "Estimation of Response Functions Based on Variational Bayes Algorithm in Dynamic Images Sequences" was retracted in 2017. Reasons: plagiarism; duplicate publication; overlap with other authors' work; overlap with earlier publications.

In this paper, we will study the probabilistic models of response functions using Bayesian methodology within the general blind source separation model [11]. The Bayesian approach was chosen for its inference flexibility and for its ability to incorporate prior information of models [12, 13]. We will formulate the prior model for general blind source separation problem with deconvolution [10] where the hierarchical structure of the model allows us to study various versions of prior models of response functions. Specifically, we design different prior models of the response functions with more parameters than the number of points in the unknown response function. The challenge is to regularize the estimation procedure such that all parameters are estimated from the observed data. We will use the approximate Bayesian approach known as the variational Bayes method [14]. The resulting algorithms are tested on synthetic as well as on real datasets.

## 2. Probabilistic Model of Image Sequences

A probabilistic model of image sequences is introduced in this section. Estimation of the model parameters yields an algorithm for Blind Source Separation and Deconvolution. Prior models of all parameters except for the response functions are described here while the priors for the response functions will be studied in detail in the next section.

### 2.1. Model of Observation

Each recorded image is stored as a column vector **d**_*t*_ ∈ **R** ^*p*×1^, *t* = 1,…, *n*, where *n* is the total number of recorded images. Each vector **d**_*t*_ is supposed to be an observation of a superposition of *r* source images a_*k*_ ∈ **R** ^*p*×1^, *k* = 1,…, *r*, stored again columnwise. The source images are weighed by their specific activities in time *t* denoted as $x_{1,t},\ldots ,x_{r,t}\equiv {\overset{-}{x}}_{t}\in R^{1\times r}$. Formally,

(1) $$\begin{array}{c} d_{t}\in a_{1}x_{1,t}+a_{2}x_{2,t}+\cdots +a_{r}x_{r,t}+e_{t}=A{\overset{-}{x}}_{t}^{T}+e_{t}, \end{array}$$

where e_*t*_ is the noise of the observation, *A* ∈ **R** ^*p*×*r*^ is the matrix composed of source images as its columns *A* ∈ [a_1_,…, a_*r*_], and symbol ()^*T*^ denotes transposition of a vector or a matrix. Equation (1) can be rewritten in the matrix form. Suppose that the observation matrix *D* = [d_1_,…, d_*n*_] ∈ **R** ^*p*×*r*^ and the matrix with TACs in its columns $X=[{\overset{-}{x}}_{1}^{T},\ldots ,{\overset{-}{x}}_{1}^{T}{]}^{T}\in R^{n\times r}$. Note that we will use the bar symbol, ${\overset{-}{x}}_{k}^{}$, to distinguish the *k*th row of matrix *X*, while *x*_*k*_ will be used to denote the *k*th column. Then, (1) can be rewritten into the matrix form as

(2) $$\begin{array}{c} D=AX^{T}+E. \end{array}$$

The tracer dynamics in each compartment is commonly described as convolution of common input function, vector *b* ∈ **R** ^*n*×1^, and source-specific response function (convolution kernel, mathematically), vector **u**_*k*_ ∈ **R** ^*n*×1^, *k* = 1,…, *r* [5, 6, 15]. Using convolution assumption, each TAC can be rewritten as

(3) $$\begin{array}{c} x_{k}=Bu_{k},\;\forall k=1,\ldots ,r, \end{array}$$

where the matrix *B* ∈ **R** ^*n*×*n*^ is composed of elements of input function *b* as

(4) $$\begin{array}{c} B=\left(\begin{array}{cccc} b_{1} & 0 & 0 & 0\\ b_{2} & b_{1} & 0 & 0\\ \cdots & b_{2} & b_{1} & 0\\ b_{n} & \cdots & b_{2} & b_{1} \end{array}\right). \end{array}$$

Suppose that the aggregation of response function *U* = [**u**_1_,…, **u**_*r*_] ∈ **R** ^*n*×*r*^. Then, *X* = *BU* and model (2) can be rewritten as

(5) $$\begin{array}{c} D=AU^{T}B^{T}+E. \end{array}$$

The task of subsequent analysis is to estimate the matrices *A* and *U* and the vector *b* from the data matrix *D*.

The article "Estimation of Response Functions Based on Variational Bayes Algorithm in Dynamic Images Sequences" was retracted in 2017. Reasons: plagiarism; duplicate publication; overlap with other authors' work; overlap with earlier publications.

### 2.2. Noise Model

We assume that the noise has homogeneous Gaussian distribution with zero mean and unknown precision parameter *ω*, *e*_*i*,*j*_ = *𝒩*_*e*_*i*,*j*__(0, *ω* ^−1^). Then, the data model (2) can be rewritten as

(6) $$\begin{array}{c} f\left(\;D\;|\;A,X,\omega \;\right)=\overset{n}{\underset{t=1}{\prod }}N_{d_{t}}\left(\;A{\overset{-}{x}}_{t},\omega^{-1}I_{p}\;\right), \end{array}$$

where symbol *𝒩* denotes Gaussian distribution and *I*_*p*_ is identity matrix of the size given in its subscript. Since all unknown parameters must have their prior distribution in the variational Bayes methodology, the precision parameter (inverse variance) *ω* has a conjugate prior in the form of the Gamma distribution

(7) $$\begin{array}{c} f\left(\;\omega \;\right)=G_{\omega }\left(\;\vartheta_{0},\rho_{0}\;\right) \end{array}$$

with chosen constants shape parameter *ϑ*_0_ and scale parameter *ρ*_0_, due to the homogeneous noise model.

The article "Estimation of Response Functions Based on Variational Bayes Algorithm in Dynamic Images Sequences" was retracted in 2017. Reasons: plagiarism; duplicate publication; overlap with other authors' work; overlap with earlier publications.

### 2.3. Probabilistic Model of Source Images

The only assumption on source images is that they are sparse; that is, only some pixels of source images are nonzeros. The sparsity is achieved using prior model that favors sparse solution depending on data [16]. We will employ the automatic relevance determination (ARD) principle [17] based on joint estimation of the parameter of interest together with its unknown precision. Specifically, each pixel *a*_*i*,*j*_ of each source image has Gaussian prior truncated to positive values (see Appendix A.1) with unknown precision parameter *ξ*_*i*,*j*_ which is supposed to have conjugate Gamma prior as

(8) fai,k ∣ ξi,k=tNai,j0,ξi,k−1,fξi,k=Gξi,kϕ0,ψ0

for ∀*i* = 1,…, *p*, ∀*k* = 1,…, *r*, and *ϕ*_0_, *ψ*_0_ are chosen constants. The precisions *ξ*_*i*,*j*_ form the matrix Ξ of the same size as *A*.

### 2.4. Probabilistic Model of Input Function

The input function **b** is assumed to be a positive vector; hence, it will be modeled as truncated Gaussian distribution to positive values with scaling parameter *ς* ∈ **R** as

(9) fb ∣ ς=tN0n,1,ς−1In,fς=Gζ0,η0,

where 0_*n*,1_ denotes zeros matrix of the given size and *ζ*_0_, *η*_0_ are chosen constants.

### 2.5. Models of Response Functions

So far, we have formulated the prior models for source images *A* and input function **b** from decomposition of the matrix *D*. The task of this paper is to propose and study prior models for response functions *U* as illustrated in Figure 1. Different choices of the priors on the response functions have strong influence on the results of the analysis which will be studied in the next section.

## 3. Nonparametric Prior Models of Response Function

Here, we will formulate several prior models of response functions. Our purpose is not to impose any parametric form as it was done, for example, in [5, 6], but to model response function as a free-form curve with only influence from their prior models. The motivation is demonstrated in Figure 2, where a common parametric model [6] is compared to an example of response function obtained from real data. While the basic form of the response function is correct, exact parametric form of the function would be very complex. Therefore, we prefer to estimate each point on the response function individually. However, this leads to overparameterization and poor estimates would result without regularization. All models in this section introduce regularization of the nonparametric function via unknown covariance of the prior with hyperparameters.

### 3.1. Orthogonal Prior

The first prior model assumes that each response function **u**_*k*_, *k* = 1,…, *r*, is positive and each response function is weighed by its own precision relevance parameter *v*_*k*_ ∈ **R** which has a conjugate Gamma prior:

(10) fuk ∣ vk=tNuk0n,1,vk−1In,fvk=Gvkα0,β0

for ∀*k* = 1,…, *r* and where *α*_0_, *β*_0_ are chosen constants.

The article "Estimation of Response Functions Based on Variational Bayes Algorithm in Dynamic Images Sequences" was retracted in 2017. Reasons: plagiarism; duplicate publication; overlap with other authors' work; overlap with earlier publications.

The precision parameters *v*_*k*_ serve for suppression of weak response functions during iterative computation and therefore as parameters responsible for estimation of the number of relevant sources.

### 3.2. Sparse Prior

The model with sparse response functions has been introduced in [10]. The key assumption of this model is that the response functions are most likely sparse which is modeled similarly as in case of source images, Section 2.2, using the ARD principle. Here, each element of response function *u*_*k*,*j*_ has its relevance parameter *v*_*k*,*j*_ which is supposed to be conjugate Gamma distributed. In vector notation, each response function **u**_*k*_ has its precision matrix *Υ*_*k*_ with precision parameters *v*_*k*,*j*_ on its diagonal and zeros otherwise. Then

(11) fuk ∣ Υk=tNuk0n,1,Υk,fvk,j=Gvk,jα0,β0,∀j=1,…,n,

where *α*_0_, *β*_0_ are chosen constants.

The employed ARD principle should suppress the noisy parts of response functions which should lead to clearer response functions and subsequently to clearer TACs.

### 3.3. Wishart Prior

So far, we have modeled only the first or the second diagonal of the precision matrix *Υ*_*k*_. Each of these approaches has its advantages which we would like to generalize into estimation of several diagonals of the prior covariance matrix. However, this is difficult to solve analytically. Instead, we note that it is possible to create the model for the full prior covariance matrix of the response functions as well as their mutual interactions. For this task, we use vectorized form of response functions denoted as **u** ∈ **R** ^*nr*×1^, **u** = vec(*U*) = [**u**_1_^*T*^,…, **u**_*r*_^*T*^]^*T*^. This rearranging allows us to model mutual correlation between response functions. The full covariance matrix *Υ* ∈ **R** ^*nr*×*nr*^ can be modeled as follows:

(12) fu ∣ Υ=tNu0nr,1,Υ−1,fΥ=WΥα0Inr,β0,

where *𝒲* is the Wishart distribution with parameters *α*_0_, *β*_0_. See Appendix A.2.

The advantage of this parameterization is obvious: the full covariance matrix is estimated. The disadvantage in this model is that, for estimation of *nr* parameters in vector **u**, we need to estimate *n* ^2^ *r* ^2^ additional parameters in covariance structure. The problem is regularized by the prior on *Υ*, which is relatively weak regularization with potential side effects. We try to suppress these side effects in the next section.

### 3.4. Variational Bayes Approximate Solution

The whole probabilistic model comprises (6)-(7), (8), and (9) and selected response functions model from Sections 3.1–3.3. The probabilistic model is solved using variational Bayes (VB) method. Here, the solution is found in the form of probability densities of the same type of the priors. The shaping parameters of the posterior densities form a set of implicit equations, Appendix B, which is typically analytically intractable and has to be solved iteratively.

The article "Estimation of Response Functions Based on Variational Bayes Algorithm in Dynamic Images Sequences" was retracted in 2017. Reasons: plagiarism; duplicate publication; overlap with other authors' work; overlap with earlier publications.

The algorithms are summarized in Algorithm 1. We named our algorithms as Nonparametric Variational Bayes Approximation (NVBA) algorithm. All prior parameters are set to 10^−10^ or 10^+10^ in order to obtain noninformative priors. The initial response functions are selected as pulses with different lengths with respect to covering the typical structures while the initial input function is selected as an exponential curve since the iterative solution could converge only to a local minimum.

**Algorithm 1 (iterative NVBA algorithm).**

(1) Initialization:
  (a) Set prior parameters *α*_0_, *β*_0_, *ϑ*_0_, *ρ*_0_, *ϕ*_0_, *ψ*_0_, *ζ*_0_, *η*_0_.
  (b) Set initial values for $\hat{A}$, $\hat{A^{T}A}$, $\hat{\Xi }$, $\hat{u}$, $\hat{u^{T}u}$, $\hat{\Upsilon }$, $\hat{b}$, $\hat{b^{T}b}$, $\hat{\varsigma }$, $\hat{\omega }$.
  (c) Set the initial number of sources  *r*_max_.
(2) Iterate until convergence is reached using computation of shaping parameters from Appendix B:
  (a) Source images $\mu_{{\overset{-}{a}}_{i}}$, $\Sigma_{{\overset{-}{a}}_{i}}$ and their variances *ϕ*_*i*_, *ψ*_*i*_, ∀*i* using (B.1)–(B.4).
  (b) Response functions *μ*_**u**_, Σ_**u**_ and their hyperparameters depending on version of the prior:
    (i) OrthogonalRF: (B.11) and (B.12),
    (ii) SparseRF: (B.11) and (B.13),
    (iii) WishartRF: (B.11) and (B.14).
  (c) Input function *μ*_**b**_, Σ_**b**_ and its variance *ζ*, *η* using (B.5)–(B.7).
  (d) Variance of noise *ϑ*, *ρ* using (B.8)–(B.9).
(3) Report estimates of source images $\hat{A}$, response functions $\hat{U}$, and input function $\hat{b}$.

## 4. Experiments and Discussion

We proposed three versions of model of nonparametric response functions within the model of probabilistic blind source separation model in Sections 3.1–3.3. The proposed algorithms are tested on simulated phantom study as well as on representative clinical data set from dynamic renal scintigraphy.

### 4.1. Synthetic Dataset

Performance of the proposed models of response functions is first studied on a synthetic dataset generated according to model (5). The size of each image is 50 × 50 pixels and the number of simulated time points is *n* = 50. We simulate 3 sources which are given in Figure 3, top row, using their source images and response functions together with generated input function **b** (top row, right). We generate homogeneous Gaussian noise with standard deviation 0.3 of the signal strength.

The article "Estimation of Response Functions Based on Variational Bayes Algorithm in Dynamic Images Sequences" was retracted in 2017. Reasons: plagiarism; duplicate publication; overlap with other authors' work; overlap with earlier publications.

The results of the three proposed models are given in Figure 3 in the rowwise schema. Note that all algorithms are capable of estimating the correct number of sources. It can be seen that all methods estimated the source images correctly. The main differences are in estimated response functions, the fourth to the sixth columns, and estimated input function, the seventh column. Note that only the first prior, orthogonal, was not able to respect the sparse character of the modeled response functions; all other priors were able to do so.

### 4.2. Competing Methods

There are some other methods which provide solution to estimate the response functions in a nonparametric fashion as well.

1. *FIR Filter.* A semiparametric approach based on finite impulse response filter (FIR Filter) is used to model the haemodynamic response functions [9].
2. *S-BSS-vecDC.* The sparse blind source separation and vectorized deconvolution (S-BSS-vecDC) algorithm is used in hierarchical models [10].

Quality of estimation of the proposed methods is validated with quantitative results using mean square error (MSE). Here the MSE (*μ*_MSE_^*k*^) is computed between the estimated response functions ${\hat{U}}_{j}$ and their simulated values *U*_*j*_^sim^:

(13) $$\begin{array}{c} \mu_{MSE}^{k}=\frac{1}{n}\overset{n}{\underset{j=1}{\sum }}{\left(\;{\hat{U}}_{j,k}-U_{j,k}^{sim}\;\right)}^{2}. \end{array}$$

*k* = 1,…, 4 is the set number of testing image. We compare the estimation results of the FIR filter, S-BSS-vecDC, and our NVBA with Wishart Prior with 4 sets of images [18].  Figure 4 gives the bar figure of Table 1.

For the four sets of images, the proposed NVBA with Wishart prior algorithm provided the best estimate of the response function (in terms of the MSE).

### 4.3. Datasets from Dynamic Renal Scintigraphy

The methods from Sections 3.1–3.3 were tested on real data from dynamic renal scintigraphy taken from online database (http://www.dynamicrenalstudy.org/). We illustrate the possible outcome of the method on two distinct datasets, numbers 84 and 42. Each dataset represents different behavior of the methods.

Both sequences consist of 50 frames taken after 10 seconds and both were preprocessed by selection region of the left kidney. The data are expected to contain three sources of activity: (i) parenchyma, the outer part of a kidney where the tracer is accumulated at the first, (ii) pelvis, the inner part of a kidney where the accumulation has physiological delay, and (iii) background tissues which is typically active at the beginning of the sequence. Since the noise in scintigraphy is Poisson distributed, the assumption of homogeneous Gaussian noise (6) can be achieved by asymptotic scaling known as the correspondence analysis [19] which transforms the original data *D*_orig_ as

(14) $$\begin{array}{c} d_{ij}=\frac{d_{ij,orig}}{\sqrt{\sum_{i=1}^{p}d_{ij,orig}\sum_{j=1}^{n}d_{ij,orig}}}. \end{array}$$

First, we applied the methods from Sections 3.1–3.3 on dataset number 84 as a typical noncontroversial case. The results are shown in Figure 5 using the estimated source images (columns 1–3), the estimated related response functions (columns 4–6), and the estimated input function (column 7). The results of all three methods are comparable with the main difference being in the smoothness or nonsmoothness of the estimated response functions. This is most remarkable in the fifth column corresponding to the response functions of the pelvis. The sparse prior prefers sparse solution with many zeros, while the Wishart prior models full covariance of response function where no smoothness is incorporated. However, the differences in this case are relatively minor. Second, we apply the methods 3.1–3.3 on dataset number 42 where different methods yield more distinct results; see Figure 6. Note that the sparse priors were not able to separate the pelvis which is mixed with the parenchyma in the first column while the orthogonal prior estimated the source images reasonably; however, the response functions of the parenchyma and the pelvis are clearly mixed. The Wishart prior was able to separate the parenchyma and the pelvis correctly together with meaningful estimates of their response functions. In this case, the use of more complex prior models significantly outperformed the simpler models. Indeed, the analysis of the full database would be of interest in concrete application; however, it is not a goal of this paper.

The article "Estimation of Response Functions Based on Variational Bayes Algorithm in Dynamic Images Sequences" was retracted in 2017. Reasons: plagiarism; duplicate publication; overlap with other authors' work; overlap with earlier publications.

## 5. Conclusion

A common model in functional analysis of dynamic image sequences assumes that the observed images arise from superposition of the original source images weighed by their time-activity curves. Each time-activity curve is assumed to be a result of common input function and source-specific response function, both unknown. Estimation of the model parameters yields an algorithm for blind source separation and deconvolution. The focus of this study is the prior model of the response functions while the models of the source images and the input function are the same. We propose three prior models of the response functions. The advantage of all three models is their flexibility in estimation of various shapes of response functions since we do not impose any parametric form of them. The formulated probabilistic models in the form of hierarchical priors are solved using the variational Bayes methodology. The performance of the proposed methods is tested on simulated dataset as well as on representative real datasets from dynamic renal scintigraphy. It is shown that the behaviors of the methods well correspond with their prior expectations. We compared our algorithm with the other competing methods, and our method achieved the most accurate result. We conclude that the most complex model, that is, the Wishart model, provides also the most desirable results in the sense of mean square errors to the original simulated data as well as in sense of biologically meaningfulness of the results on the real datasets. Notably, the methods have no domain-specific assumptions; hence, they can be used in other tasks in dynamic medical imaging.

## Figures and Tables

**Figure 1:** Hierarchical model for image sequences.

**Figure 2:** Example of theoretical shape of response function (by [6]), left, and corresponding real-world shape of convolution kernels, right.

**Figure 3:** The results of the three studied methods on synthetic dataset (the first row). The red lines are generated data while the blue lines are estimated results from the respective methods.

**Figure 4:** Comparison of MSE of response functions with different sets of images.

**Figure 5:** Estimated source images (columns 1–3), response functions (columns 4–6), and input functions (column 7) using priors: orthogonal, sparse, and Wishart.

**Figure 6:** Estimated source images (columns 1–3), response functions (columns 4–6), and input functions (column 7) using priors: orthogonal, sparse, and Wishart.

**Table 1:** Comparison of MSE of response functions with different sets of images.

Algorithm	*k*	*μ*_MSE_^*k*^
FIR filter	1	0.044
	2	0.0214
	3	0.115
	4	0.234

S-BSS-vecDC	1	0.0057
	2	0.0021
	3	0.2401
	4	0.4722

NVBA with Wishart prior	1	0.003
	2	0.0016
	3	0.0077
	4	0.0056

## Appendix

### A. Required Probability Distributions

#### A.1. Truncated Normal Distribution

Truncated normal distribution, denoted as *t𝒩*, of a scalar variable *x* on interval [*a*; *b*] is defined as

(A.1) $$\begin{array}{c} tN\left(\;\mu ,\sigma \left[\;a,b\;\right]\;\right)=\frac{\sqrt{2}\exp\left({\left(x-\mu \right)}^{2}\right)}{\sqrt{\pi \sigma }\left(erf\left(\beta \right)-erf\left(\alpha \right)\right)}\chi_{\left[a,b\right]}\left(\;x\;\right), \end{array}$$

where $\alpha =\left(a-\mu \right)/\sqrt{2\sigma }$, $\beta =\left(b-\mu \right)/\sqrt{2\sigma }$, function *χ*_[*a*, *b*]_(*x*) is a characteristic function of interval [*a*, *b*] defined as *χ*_[*a*, *b*]_(*x*) = 1 if *x* ∈ [*a*, *b*], and *χ*_[*a*, *b*]_(*x*) = 0 otherwise. erf() is the error function defined as $erf\left(t\right)=\left(2/\sqrt{\pi }\right)\int_{0}^{t}e^{-u^{2}}du$.

The article "Estimation of Response Functions Based on Variational Bayes Algorithm in Dynamic Images Sequences" was retracted in 2017. Reasons: plagiarism; duplicate publication; overlap with other authors' work; overlap with earlier publications.

The moments of truncated normal distribution are

(A.2) x^=μ−σ2exp⁡−β2−exp⁡−α2πσerfβ−erfα,x2^=σ+μx^−σ2b exp−β2−a exp−α2πerfβ−erfα.

#### A.2. Wishart Distribution

Wishart distribution *𝒲* of the positive-definite matrix *X* ∈ **R** ^*p*×*p*^ is defined as

(A.3) WpΣ,vXv−p−1/22−vp/2Σ−v/2Γp−1v2·exp⁡−12trΣ−1X,

where Γ_*p*_(*v*/2) is the Gamma function. The required moment is

(A.4) $$\begin{array}{c} \hat{X}=v\Sigma . \end{array}$$

### B. Shaping Parameters of Posteriors

Shaping parameters of posterior distributions are given as

(B.1) Σa−i=ω^∑j=1nx−jTx−j^+diagΞi^−1,

(B.2) μa−i=Σa−iω^∑j=1nx−j^di,j,

(B.3) ϕi=ϕi,0+121r,1,

(B.4) ψi=ψi,0+12diaga−iTa−i^,

(B.5) Σb=ς^In+ω∑i,j=1ra−jTa−j^∑k,l=0n−1ΔkTΔluk+1,jul+1,i^−1,

(B.6) μb=Σbω^∑k=1r∑j=0n−1Δjuj+1,k^TDTak^,

(B.7) ζ=ζ0+n2,

(B.8) ϑ=ϑ0+np2,

(B.9) ρ=ρ0+12trDDT−A^D^TDT−DX^TA^T+12trATA^XTX^.

Here, $\hat{x}$ denotes a moment of respective distribution, tr() denotes a trace of argument, diag() denotes a square matrix with argument vector on diagonal and zeros otherwise or a vector composed from diagonal element of argument matrix, and 1_*n*,1_ denotes the matrix of ones of dimension *n* × 1; the auxiliary matrix Δ_*k*_ ∈ **R** ^*n*×*n*^ is defined as

(B.10) $$\begin{array}{c} {\left(\;\Delta_{k}\;\right)}_{i,j}=\left\{\begin{array}{cc} 1, & \text{if}\;\;i-j=k\\ 0, & \text{otherwise,} \end{array}\right. \end{array}$$

and standard moments of required probability distributions are given in Appendices A.1 and A.2.

The shaping parameters for response functions are given in the following subsections while the parameter *μ*_**u**_ is common for all methods as

(B.11) μu=ΣuATA^⊗ω^BTB^vecBTB^−1B^TDTA^ATA^−1.

#### B.1. Shaping Parameters for Orthogonal Prior

Consider

(B.12) Σu=ATA^⊗ω^BTB^+In⊗Υ^−1,αk=αk,0+n2,βk=βk,0+12trukukT.

#### B.2. Shaping Parameters for Sparse Prior

Consider

(B.13) Σu=ATA^⊗ω^BTB^+diagvecΥ^−1,α=α0+121nr,1,β=β0+12diaguuT^.

#### B.3. Shaping Parameters for Wishart Prior

Consider

(B.14) Σu=ATA^⊗ω^BTB^+Υ^−1,ΣΥ=uuT^+α0Inr−1−1,β=β0+1.
